This article has been retracted.

# Computerized misinterpretation of QT interval in 12‐lead electrocardiogram and its clinical consequences: A case of recurrent syncope

**DOI:** 10.1002/joa3.12817

**Published:** 2023-01-30

**Authors:** Kanae Hasegawa, Yoshitomo Fukuoka, Seiko Ohno, Minoru Horie, Hiroshi Tada

**Affiliations:** ^1^ Department of Cardiovascular Medicine, Faculty of Medical Sciences University of Fukui Fukui Japan; ^2^ Department of Bioscience and Genetics National Cerebral and Cardiovascular Center, Suita Osaka Japan; ^3^ Department of Cardiovascular Medicine Shiga University of Medical Science Otsu Shiga Japan

**Keywords:** automated diagnosis, long QT syndrome, QT interval, syncope

## Abstract

Don't blindly accept the automated assessment of electrocardiogram. It is important to raise long QT syndrome to the differential diagnosis of repeated syncope.

A 27‐year‐old female visited our emergency room in the middle of the night because she experienced syncope several times throughout the preceding 2 days upon waking up and when attempting to walk at night. At the time of the visit, her consciousness level was clear and plasma potassium concentration was 4.0 mEq/L (normal range: 3.6–4.8 mEq/L). Her 12‐lead electrocardiogram (ECG) revealed sinus rhythm (65 beats/min) and QT prolongation with low amplitude T waves (QT/QTc [intervals], 600/640 ms) (Figure 1A). Echocardiography, chest X‐ray, and brain magnetic resonance imaging (MRI) findings were normal. She was admitted for follow‐up due to the presence of marked QT prolongation on 12‐lead ECG. Five hours after the admission, torsades de pointes (TdP) spontaneously occurred with typical initiating “short‐long‐short” sequences (Figure 1B) when she felt faint. She had no abnormal ECG findings in past school physical examinations. She had no family history of syncope, sudden death, or long QT syndrome (Figure 2A). ECGs of her mother and son showed no QT prolongation (Figure 2A).

**FIGURE 1:** (A) Twelve‐lead electrocardiogram on admission. (B) Tracings of bedside continuous single‐lead ECG after admission. Torsades de pointes spontaneously occurred with typical initiating the “short‐long‐short” sequence.

**FIGURE 2:** (A) Pedigree of KCNH2, (P).R176fsX331. Circles and squares indicate females and males, respectively. Closed symbol indicates a history of syncope. Plus signs indicate variant positive subjects, whereas minus signs indicate variant negative subjects. The black arrow indicates the proband of the family. Electrocardiograms in lead V5 of the patient's mother and son showed no QT prolongation. (B) Electropherograms of *KCNH2* in control and the *KCNH2* gene variant, p.R176fsX331(c. 526dupC), in the patient.

A detailed medical history revealed that she experienced nightmares during sleep, which were followed by convulsions and groaning, at the age of 19. She fainted twice after waking up in the morning. The patient visited a neurology clinic and underwent a brain MRI, but the underlying cause remained unknown. At the age of 21, she experienced dizziness while walking or trying to get up in the morning. She experienced syncope and visited a hospital, where automated ECG diagnosis was within the normal range (Figure 3A,B). Brain computed tomography and electroencephalogram revealed no obvious abnormality. Therefore, the physician found no apparent cause for her syncope, and she returned home. The patient continued to have episodes of syncope several times a year until she was 27. Throughout this period, she visited several hospitals and clinics. However, episodes of syncope due to long QT syndrome were not suspected, and the patient did not undergo another ECG examination nor was referred to a cardiologist.

**FIGURE 3:** (A) Twelve‐lead electrocardiogram (ECG) recorded when the patient was aged 21 years. The manually measured QT/QTc intervals were 580/608 ms. (B) An automated diagnosis based on ECG.

After admission to our hospital, the ECG recorded at the age of 21 was retrieved and reevaluated. Her ECG revealed QT prolongation with notched T waves (Figure 3A), a finding that was clearly abnormal (QT/QTc, 580/608 ms). Genetic analysis for long QT syndrome, including *KCNQ1*, *KCNH2*, *SCN5A*, *KCNE1*, and *KCNE2* was performed after obtaining written informed consent from the patient. A novel frameshift variant that resulted from duplication (c. 526dupC, p.R176fsX331) in *KCNH2* was identified (Figure 2B). Her mother and son, who did not have QT prolongation, did not carry the variant (Figure 2A).

The patient was diagnosed with type 2 long QT syndrome. Carvedilol was initiated at 5.0 mg per day, and the dose was gradually increased. One month later, her QT interval had shortened (QT/QTc, 480/488 ms), and notched T waves had disappeared (Figure 4A). After 6 months of receiving 10 mg carvedilol per day, her QT interval completely normalized (QT/QTc, 450/442), and T‐wave shape was no longer abnormal (Figure 4B). The patient recovered well, and no syncope recurrence was observed throughout a 3‐year follow‐up period.

**FIGURE 4:** Twelve‐lead electrocardiograms after daily oral administration of (A) 5, and (B) 10 mg carvedilol.

## 1 DISCUSSION

This report describes a case of recurrent episodes of syncope that persisted for 8 years. When initial 12‐lead ECG findings were obtained, the physician did not evaluate the data carefully. Instead, the physician relied on an automated ECG diagnosis that was obtained using ECG analysis software. After the QT interval in the patient's 12‐lead ECG was first misinterpreted via an automated ECG diagnosis, no physicians recommended a repeat ECG examination or reviewed prior findings, despite the recurrence of syncope episodes.

Cardiac syncope is the second most common type of syncope,^1^ and arrhythmias, including TdP, are its most common cause.^2^ Moreover, patients with cardiac syncope have the highest risk of recurrence and are at increased risk of death from any cause related to syncope.^1^ ECG facilitates the diagnosis of cardiac syncope and improves the prognosis of patients. Therefore, to ensure an accurate diagnosis and determine the cause of syncope, multiple ECG examinations and careful analysis of the results are crucial.^2^ Automated ECG diagnosis benefits physicians because it reduces the effort needed to evaluate ECG findings and allows physicians to immediately use findings in the clinic. The automated ECG diagnoses are widely utilized in medical practices with non‐expert physicians and medical staff.^3^ However, automated ECG diagnoses are not always correct. In particular, QT prolongation is underestimated or unreported via diagnostic software,^4^ and measurement differences between algorithms in the determination of QT interval are larger in patients with congenital and acquired long QT intervals than in healthy subjects. A previous study revealed that automated ECG diagnosis concluded that findings were “normal” in 42.1% of patients with a prolonged QTc interval.^4^ The phenomenon was observed for algorithms from various manufacturers. From these perspectives, automated ECG diagnosis plus over‐reading by physicians offer the accurate diagnosis, and long QT syndrome experts strongly advocate manual measurement.^5^

In the present case, apparent and obvious QT prolongation at 21 years of age (Figure 3A) was missed due to an incorrect automated ECG diagnosis. T waves in leads I, II, III, aVR, aVF, and V2‐V6 had prominent notches, and the second component of the T wave should have been included in the analysis of the QT interval.^5^ The automated ECG diagnosis did not consider the second component of the notched T wave and instead regarded the endpoint of the first component of the notched T wave as the endpoint of the QT interval. If the physician had self‐evaluated ECG findings, they would have noticed the markedly prolonged QT interval and bimodal T waves, even if the QT interval was inaccurately measured.

## CONFLICT OF INTEREST

There are no conflicts of interest.

## APPROVAL OF THE RESEARCH PROTOCOL

Research Ethics Committee of University of Fukui (No. 20200027).

## INFORMED CONSENT

The patient provided informed consent.

## REGISTRY AND THE REGISTRATION NO. OF THE STUDY/TRIAL

N/A.

## ANIMAL STUDIES

N/A.
